# SIRT3 regulates cell proliferation and apoptosis related to energy metabolism in non-small cell lung cancer cells through deacetylation of NMNAT2

This article has been retracted.

**DOI:** 10.3892/ijo.2013.2103

**Published:** 2013-09-16

**Authors:** HONGQI LI, ZHIQIANG FENG, WEIZHANG WU, JING LI, JINQIAN ZHANG, TINGYI XIA

**Affiliations:** 1 Department of Radiation Oncology, Air Force General Hospital, Beijing 100142;; 2 Department of Radiation Oncology, Daping Hospital, The Third Military Medical University, Chongqing 400030;; 3 Institute of Infectious Diseases, Beijing Ditan Hospital, Capital Medical University, Beijing 100015;; 4 Department of Radiation Oncology, The General Hospital of Chinese People’s Liberation Army, Beijing 100853, P.R. China

**Keywords:** SIRT3 protein, energy metabolism, lung neoplasms, acetylation, NMNAT2 protein

## Abstract

Lung cancer is the leading cause of death worldwide and associated with dismal prognoses. As a major mitochondrial deacetylase, SIRT3 regulates the activity of enzymes to coordinate global shifts in cellular metabolism and has important implications for tumor growth. Its role as a tumor suppressor or an oncogene in lung cancer is unclear, especially in non-small cell lung carcinoma (NSCLC). To identify the mechanism of SIRT3-interacting proteins, we performed a yeast two-hybrid screen using a human lung cDNA library. One of the positive clones encoded the full-length cDNA of the nicotinamide mononucleotide adenylyltransferase 2 (NMNAT2) gene and the interaction between SIRT3 and NMNAT2 was identified. The interaction on growth, proliferation, apoptosis of NSCLC cell lines, and energy metabolism related to SIRT3 were investigated. Screening from the library resulted in NMNAT2 gene. We found that NMNAT2 interacts with SIRT3 both *in vitro* and *in vivo*; SIRT3 binds to NMNAT2 deacetylating it. Downregulation of SIRT3 inhibited acetylation of NMNAT2 and NAD^+^ synthesis activity of the enzyme. Low expression of SIRT3 significantly inhibited mitotic entry, growth and proliferation of NSCLC cell lines and promoted apoptosis, which was related to energy metabolism involving in the interaction between SIRT3 and NMNAT2. Taken together, our results strongly suggest that the binding of SIRT3 with NMNAT2 is a novel regulator of cell proliferation and apoptosis in NSCLC cell lines, implicating the interaction between SIRT3 and NMNAT2, energy metabolism associated with SIRT3.

## Introduction

Lung cancer is the most common cause of cancer deaths worldwide, ∼1.2 million deaths people die from it per year (1). It is the leading type of new cancer cases leading to death (2). Non-small cell lung carcinoma (NSCLC) is the most frequent subtype, ∼85% of all cases. Most of NSCLC patients have locally advanced or distant metastatic disease (stage III/IV) from onset of symptoms. It is strongly associated with poor prognosis and has a 5-year survival rate of <10 and 5% in male and female patients, respectively (3). Platinum-doublet regimen remains the standard with modest survival benefits, although also improved response rates (RRs) have been reported. However, the RRs is ranging from 17 to 32% and progression-free survival (PFS) of 3.1–5.5 months, overall survival (OS) of 7.4–11.3 months (4–7). To improve clinical outcome for patients with lung cancer, targeted therapies are increasingly being used, particularly in patients with specific molecular features.

Altered metabolism is a hallmark of tumor cells supporting rapid cell proliferation (8). Many metabolic intermediates that support cell growth are provided by mitochondria; consequently, there is great interest in elucidating how mitochondrial metabolic pathways are regulated. The role of the conserved sirtuin family of deacetylases in nutrient-sensitive regulation of metabolic pathways is important, especially on the mitochondrial sirtuin, SIRT3. By deacetylating proteins involved in multiple mitochondrial processes, SIRT3 can co-ordinate global shifts in mitochondrial activity, with important implications for tumor growth (9).

The vision of Warburg on cancer cell metabolism, that sidelined mitochondria as dysfunctional bystanders, must be revised. It includes the critical contribution of mitochondria supporting tumor growth. The main function of the mitochondrion is the production of energy, in the form of adenosine triphosphate (ATP). ATP from non-proliferating cells are rewired to serve as biosynthetic factories in rapidly proliferating cells and SIRT3 could serve as an important regulator of the balance between glycolytic and anabolic pathways and mitochondrial oxidative metabolism to regulate tumor cell growth (9,10). In nutrient-deprived conditions, SIRT3 deacetylates numerous mitochondrial proteins to promote nutrient oxidation and ATP production. Conversely, low SIRT3 activity increases ROS production, which signals through HIF1α to increase glycolytic metabolism and cellular proliferation. Increasing evidence indicates that SIRT3 plays a unique regulatory role, integrating mitochondrial regulation with intracellular signaling cascades. By targeting more than a half a dozen key metabolic enzymes, SIRT3 is perfectly positioned to orchestrate coordinated shifts in mitochondrial metabolism, with potential implications for diseases that rely on mitochondrial metabolic activities. It will be important for future studies to increase our understanding of how mammalian sirtuins integrate metabolism with signaling cascades by post-translational modification of diverse substrates and how modulation of sirtuin activity can influence health and disease (9,10). However, the role of SIRT3 as a tumor suppressor or an oncogene in lung cancer is unclear, especially in NSCLC.

Herein, to address this question, the interaction between SIRT3 and NMNAT2 and its involvement in growth, proliferation and apoptosis of NSCLC cell lines was studied. Energy metabolism associated with SIRT3 was implicated and will be further studied on the interactive mechanisms in NSCLC cell lines with the interaction and possible applications in clinical treatment for lung cancer, especially NSCLC.

## Materials and methods

### Culture cells

Human NSCLC cell lines A549, H1299 and PC-9 from ATCC were cultured in Dulbecco’s modified Eagle’s medium (DMEM) supplemented with 10% fetal bovine serum (FBS) (Gibco, USA) and 1% penicillin-streptomycinneomycin (PSN) Antibiotic Mixture (Invitrogen, USA) at 37°C in a humidified 5% CO_2_/95% air environment.

### Plasmids

For the yeast two-hybrid assay, the bait plasmid pGBKT7-SIRT3 was generated by inserting a PCR-amplified cDNA fragment containing SIRT3 into pGBKT7 (Clontech). SIRT3 was cloned into pBIND (Promega), pEGFP-C1 (Clontech), pGEX-2T vector (GE). Human full-length NMNAT2 cDNA and the cDNAs for its truncated mutants (NMNAT2 N and NMNAT2 C1–2) were PCR-amplified and subcloned in-frame into pCMV-5a (Sigma). NMNAT2 was cloned into pACT (Promega), pDsRed1-N1 (Clontech), pCDNA-3.1(−) myc/his (A) vector (Invitrogen). All plasmids were verified by restriction enzyme analysis and DNA sequencing. The hSIRT3 adenovirus was from Vector BioLabs (Philadelphia, PA, USA).

### Cell transfection and adenovirus infection

At 24–30 h after seeding, NSCLC cells were used for adenovirus infection or immunostaining as described below. The adenoviruses were used at a multiplicity of infection (MOI) of 10. Cos7 and HeLa cells were grown in Dulbecco’s modified Eagle’s medium supplemented with penicillin-streptomycin and 10% fetal bovine serum (complete growth medium). Cells were transfected with appropriate plasmids using Superfect transfection reagent (Qiagen) according to the manufacturer’s protocol. For the RNA interference experiments, NSCLC cells were transfected with 200 nM On-Target-plus small interfering RNA (siRNA) specific for hSIRT3 using Dharma-FECT transfection reagents according to the manufacturer’s protocol (11).

### Yeast two-hybrid assay

The bait plasmid pGBKT7-SIRT3 was used to screen a human lung cDNA library in pGADT7 according to the manufacturer’s instructions (Clontech). Transformants were placed on synthetic medium lacking tryptophan, leucine, adenine and histidine but containing 1 mM 3-aminotriazole. Approximately 4 million transformants were screened. The screened positive clones were also verified by one-on-one transformations and selection on agar plates lacking tryptophan and leucine, or adenine, histidine, tryptophan and leucine, respectively and were also processed by β-galactosidase assay.

### Co-immunoprecipitation

For transfection-based co-immunoprecipitation assays, cells were transfected with the indicated plasmids using Lipofectamine 2000 (Invitrogen), lysed in 0.5 ml lysis buffer (50 mM Tris at pH 8.0, 150 mM NaCl, 0.25% NP-40, 1 mM DTT and protease inhibitor tablets from Roche) and immunoprecipitated with Protein G Plus/Protein A Agarose Suspension beads (Calbiochem) for 3 h at 4°C. The beads were washed 4 times with the lysis buffer and eluted in SDS sample buffer. The eluted proteins were separated by SDS-PAGE, followed by western blotting with antibody.

### Mammalian two-hybrid analysis

To test the hypothesis of NMNAT2 interacting with SIRT3 *in vivo* using the CheckMate™ Mammalian Two-Hybrid system (Promega), plasmids pACT-NMNAT2 and plasmids pBIND-SIRT3 were constructed that were used for cotransfections of cells cultured in 6-well plates. Two micrograms of pACT-NMNAT2 plasmid and 2 *μ*g of pBIND-SIRT3 plasmid were used for cotransfections by Lipofectamine 2000. The plasmids pACT-NMNAT2+pBIND, pACT+pBIND-SIRT3, pACT, pBIND and blank were used for transfections, respectively, as a negative control. The plasmids pBIND-Id and the pACT-MyoD Control Vector were cotransfectioned as a positive control. At 48 h after transfection, cells were washed 3 times with PBS and then lysed with passive buffer. Firely luciferase assays were performed using the Dual-Glo Luciferase assay system (Promega) following the manufacturer’s instructions. The firefly results were corrected for transfection efficiency using the renilla luciferase. Significance was determined using the paired Student’s t-test on the mean of three different experiments.

### GST pull-down assay

The GST- and His-tagged fusion proteins were expressed and purified by glutathione-Sepharose 4B beads (GE) and Ni-NTA agarose (GE), respectively. The expression plasmid for NMNAT2 was used for *in vitro* transcription and translation in the TNT system (Promega). The NMNAT2 or the purified His-tagged fusion protein was incubated with GST fusion protein bound to glutathione-Sepharose beads in 0.5 ml of the binding buffer (50 mM Tris-HCl, pH 7.5, 150 mM NaCl, 1 mM EDTA, 0.3 mM DTT, 0.1% NP-40) at 4°C. The beads were precipitated, washed 4 times with the binding buffer, eluted by boiling in SDS sample buffer and analyzed by SDS-PAGE. Western blotting was performed with anti-His (Santa Cruz). A quantitative measurement of the band intensity was performed using the GE Typhoon Trio (GE, USA).

### Colocalization

Cells were grown on glass coverslips in culture plates. Cells were co-transfected with plasmids, 2 *μ*g of pEGFP-C1-SIRT3 (green fluorescent protein, GFP) and 2 *μ*g of pDS-RED1-N1- NMNAT2 by Lipofectamine™ 2000 for 48 h and then cells were treated with 4% paraformaldehyde (PFA) for 10 min, washed 3 times with PBS, stained with PBS including 0.1 *μ*g/ml 4′,6-diamidino-2-phenylindole (DAPI) for 30 min at 30°C. Confocal images were acquired using Zeiss 510 META confocal microscope.

### Western blot analyses

Western blot analyses were prepared as described (12). NSCLC cell cultures were lysed and placed in RIPA buffer (Cell signaling) with 1 mM PMSF on ice for 30 min. Cell lysates were centrifuged at 14,000 g for 10 min and cell extracts were mixed with a 1:4 volume of SDS-PAGE loading buffer (10% β-mercaptoethanol, 10% glycerol, 4% SDS, 0.01% bromophenol blue and 62.5 mM Tris-HCl, pH 6.8) and heated to 65°C for 15 min. Samples were loaded on a 10% resolving SDS-polyacrylamide gel and transferred to polyvinyldifluoridine membranes. Membranes were incubated overnight at 4°C with rabbit polyclonal anti-SIRT3 (1:500; Abcam), NMNAT2 antibody (Santa Cruz, 1:1,000 dilution), β-actin (Santa Curz, 1:1,000), GST (Santa Cruz, 1:1,000), Flag (Santa Cruz, 1:1,000), His (Santa Cruz, 1:1,000), SIRT3 (Cell Signaling, 1:1,000), Myc (Santa Cruz, 1:1,000). All affinity-purified and species-specific fluorophore-conjugated secondary antibodies were obtained from Santa Cruz and used at dilutions between 1:500 and 1:800. Immunoreactivity was detected with luminol reagent (GE).

### In vitro acetylation-deacetylation assay

Unlabeled Flag-NMNAT2 was *in vitro* translated using the TNT coupled transcription-translation rabbit reticulocyte lysate kit (Promega) and immunoprecipitated using anti-Flag M2 affinity beads. Beads with bound protein were washed 4–5 times with radioimmunoprecipitation assay buffer followed by a phosphate-buffered saline (PBS) wash. The final wash was performed in 1X HAT buffer (50 mM Tris, pH 8.0, 10% glycerol, 0.1 mM EDTA, 1 mM dithiothreitol). A typical acetylation reaction mixture contained 1 *μ*g active p300/CBP-associated factor (PCAF) enzyme (Upstate Biotechnology), 0.3 mM acetyl coenzyme A (Sigma) and 10 mM sodium butyrate in 1X HAT buffer. Reaction mixtures were incubated at 30°C for 2 h on a rotator. For the deacetylation assay, acetylated Flag-NMNAT2 that bound to the beads was washed as described above and resuspended in 1X HDAC buffer (50 mM Tris, pH 8.0, 4 mM MgCl_2_, 0.2 mM dithiothreitol). The acetylated Flag-NMNAT2 substrate was either incubated only in 1X HDAC buffer (control) or with equal amounts of Myc-SIRT3 with or without NAD (1 mM) in 1X HDAC buffer. Myc-SIRT3 catalytic was produced in a prokaryotic expression system as described (15). Reaction mixtures were incubated for 2–3 h at 37°C on a rotator. Proteins were resolved by sodium dodecyl sulfate-polyacrylamide gel electrophoresis (SDS-PAGE) and analyzed by western blotting (11).

### Cellular oxygen consumption assay

Steady state cell respiration in cells was measured in non-buffered DMEM containing 5.5 mM glucose for cells with XF^e^24 analyzer (Seahorse Bioscience) according to the manual.

### ATP production assay

Steady state cellular ATP levels were measured by using ATP bioluminescence assay kit CLS II in accordance with the protocol (Roche). The optimal detection range is between 10^−7^ and 10^−10^ M. The pH of the sample should be in the range of 7.6–8.0. ATP standard was diluted with redist water by serial dilution in the range of 10^−5^ and 10^−10^ M. Luciferase reagent was added to the samples/standards by automated injection and the measurement was started after a 1-sec delay and integrated for 1–10 sec. The blank (no ATP) was subtracted from the raw data and ATP concentrations calculated from a log-log plot of the standard curve data.

### NAD assay

NAD assay was performed as previously described (16–18). Cells were extracted in 0.5 N HClO_4_, neutralized with 3 M KOH/125 mM Gly-Gly buffer (pH 7.4) and centrifuged at 10,000 × g for 5 min. Supernatants were mixed with a reaction medium containing 0.1 mM 3-(4,5-dimethylthiazol-2-yl)-2,5-diphenyl-tetrazolium bromide (MTT), 0.9 mM phenazine methosulfate, 13 U/ml alcohol dehydrogenase, 100 mM nicotinamide and 5.7% ethanol in 61 mM Gly-Gly buffer (pH 7.4). The A560 nm was determined immediately and after 10 min and results were calibrated with NAD standards.

### Cell synchronization, BrdU labeling and mitotic index

To avoid potential carry-over effects of plasmids transfection-induced cell cycle defects in the previous cycle on the following mitotic entry during the next cycle, we transfected plasmids into cells during the interval between two thymidine blocks, so that we were able to evaluate direct impact of interaction of NMNAT2 with SIRT3 on mitotic entry (13). Cells were synchronized by double thymidine block. Briefly, cells were plated at 40% confluency and arrested with 2 mM thymidine. After 19-h incubation, cells were washed 4 times with fresh medium and treated with siRNA (NMNAT2 and control). After incubation with DNA-lipid mixture for 3 h, cells were washed twice and incubated in fresh medium for an additional 5 h. Subsequently, cells were cultured in medium containing 2 mM thymidine and 2 *μ*g/ml puromycin for the second arrest and drug selection. After 16-h incubation, cells were released into the cell cycle by incubation in fresh medium. Cells were collected or fixed at indicated time-points and subjected to specific analyses.

### BrdU labeling for evaluation of DNA synthesis

Following release from the second thymidine arrest at indicated time-points, cells grown in 12-well plate were pulse labeled with BrdU (50 *μ*M) for 30 min. After three washes of PBS, cells were fixed with 1 ml of Carnoy’s fixative (3 parts methano 1:1 part glacial acetic acid) at −20°C for 20 min and followed by three washes of PBS. Subsequently, DNA was denatured by incubation of 2M HCl at 37°C for 60 min, followed by three washes in borate buffer (0.1 M borate buffer, pH 8.5). After incubation with the blocking buffer, cells were stained with anti-BrdU antibody (BD Biosciences, 1:100) overnight at 4°C. After washes in PBS, cells were incubated with Texas Red-conjugated anti-mouse goat IgG for 30 min at RT. After washes, cells were mounted and BrdU positive cells were manually scored under immunofluorescence microscope.

Mitotic events were scored by time-lapse videomicroscopy and DNA staining. Cells were synchronized as described above. Real-time images were captured every 10 min with Openlab software. Mitotic events of cells were scored by their morphological change (from flat to round-up). For each experiment, ≥800 cells were videotaped, tracked and analyzed. Alternatively, nocodazole (100 ng/ml) was added into the medium after release, cells were collected, fixed and stained with DNA dye (Hoechst 33258). Mitotic cells were scored by nuclear morphology and DNA condensation.

### Cell growth and proliferation assay

Cell growth for 48 h was determined by the colorimetric tetrazolium derived XTT (sodium 3′-(1-(phenylaminocarbonyl)-3, 4-tetrazolium)-bis (4-methoxy-6-nitro) benzene sulfonic acid hydrate) assay (Roche Applied Science, Mannheim, Germany) and DNA synthesis of cells was assessed by the BrdU (bromodeoxyuridine) incorporation assay (Roche Applied Science). For the cell growth and proliferation assay, at 48 h after culture, the cells of each group were re-seeded in SWNHs-coated 96-well plates at a density of 0.3–1×10^4^ cells per well. After 48 h, XTT and incorporated BrdU were measured colorimetrically using a microtiter plate reader (Bio-Rad) at a wavelength of 450 nm (14).

### Cell viability assay

Cell viability was determined using a CCK-8 cell viability assay kit (Dojindo Laboratories, Japan). The cells (5×10^3^ cells/well) were pretreated with various methods as indicated and then incubated for 16 h in a 96-well plate. Cell viability assay kit solution (10 *μ*l) was added to each well of the plate. After incubation for 1 h at 37°C in the dark, absorbances were measured at 450 nm using a multi-well plate reader (15).

### Determimation of apoptosis

Apoptotic cells were identified by fluorescence-activated cell sorting (FACS) using Annexin V-Fluos (Biolegend) following the protocol of the manufacturer.

### Statistical analyses

Continuous normally distributed variables are presented as the mean ± standard deviation (SD). For statistical comparison of quantitative data between groups, analysis of variance (ANOVA) or t-test was performed. To determine differences between groups not normally distributed, medians were compared using Kruskal-Wallis ANOVA. χ^2^ test was used when necessary for qualitative data. The degree of association between variables was assessed using Spearman’s non-parametric correlation. All statistical analyses were carried out using SPSS software version 13.0 (SPSS Inc., Chicago, IL, USA). Probability values of ≤0.05 or less were considered to be statistically significant.

## Results

### Identification of NMNAT2 as a SIRT3-interacting protein by yeast two-hybrid system

To identify novel SIRT3-interacting proteins, we performed a yeast two-hybrid screening of a human lung cDNA library using full-length SIRT3 as bait. Screening of 4 million transformants resulted in the isolation of several positive clones, which were identified to encode the full-length cDNA of NMNAT2 gene. To further identify the interaction of NMNAT2 with SIRT3 in yeast, we next examined the ability of SIRT3 protein to bind to NMNAT2 in yeast cells (Fig. 1A). These data demonstrated that SIRT3 interacts with NMNAT2 in yeast cells.

### Interaction of SIRT3 with NMNAT2 in vivo and in vitro

To identify the interaction between SIRT3 and NMNAT2, we next examined the ability of SIRT3 protein to bind to NMNAT2 in mammalian cells. Cells were co-transfected with Flag-tagged SIRT3, Myc -tagged NMNAT2, or Myc control vector. Immunoprecipitation (IP) of cell lysates with an anti-Flag monoclonal antibody was followed by immunoblotting (IB) with anti-Myc. Results showed specific interaction between the Flag-SIRT3 and Myc-NMNAT2 (Fig. 1B). To test the hypothesis of SIRT3 interacting with NMNAT2 *in vivo*, the CheckMate™ Mammalian Two-Hybrid system (Promega) was used. The plasmids pACT-SIRT3 and pBIND-NMNAT2 were used for cotransfections by Lipofectamine 2000. The plasmids pACT-SIRT3+pBIND, pACT+pBIND-NMNAT2, pACT, pBIND and blank were used for transfections, respectively, as a negative control. The plasmids pBIND-Id and the pACT-MyoD Control Vector were cotransfected as a positive control. After transfection for 48 h, cells were lysed. Luciferase assays were performed using the Dual-Glo Luciferase assay system (Promega) following the manufacturer’s instructions. The results were corrected for transfection efficiency using renilla luciferase. Significance was determined using the paired Student’s t-test on the mean of three different experiments. The luciferase levels of pACT-SIRT3 and pBIND-NMNAT2 were ≥2.64 times higher than negative control (P<0.05) (Fig. 1C). The expression of SIRT3 and NMNAT2 in lysate of those cells was detected by WB with anti-SIRT3 and anti-NMNAT2 monoclonal antibody (Fig. 1D). To demonstrate the interaction of SIRT3 and NMNAT2 *in vitro*, GST pull-down assays were performed in which *in vitro* translated His-SIRT3 was incubated with full-length GST-NMNAT2 or Flag. As shown in Fig. 1E, SIRT3 interacted with GST-NMNAT2 but not with Flag alone (Fig. 1E). To test the colocalization of SIRT3 and NMNAT2 in cells, cells were grown on glass coverslips in culture plates then co-transfected with plasmids pEGFP-C1-SIRT3 and pDS-RED1-N1-NMNAT2. After 48 h, cells were stained with PFA and DAPI, confocal images were acquired using Zeiss 510 META confocal microscope. NMNAT2 (red, Fig. 1F) and SIRT3 (green, Fig. 1G) protein, all localized to the cytoplasma. The nuclear of cells (blue, Fig. 1H) were stained by DAPI. The overlaid images indicated that SIRT3 overlapped partly with NMNAT2 (Fig. 1I) in the cytoplasma. These results indicate that SIRT3 interacted with NMNAT2 *in vivo* and *in vitro*.

### Mapping of the NMNAT2 and SIRT3 interaction regions

To identify the region of SIRT3 required for its interaction with NMNAT2, Co-IP experiments were performed in which three deletion mutants. SIRT3 is cleaved by caspase-3 at two sites (D28 and D107, Fig. 2A). As shown in Fig. 2A, both full-length and the carboxy-terminal fragments of SIRT3 C1 protein interacted with Myc-NMNAT2, but the amino-terminal fragment of SIRT3 (SIRT3N, residues 1–28) did not interact with NMNAT2 (Fig. 2A). As shown in Fig. 2B, the Flag-SIRT3 C1 (29–307) bound specifically to NMNAT2, but the Flag-N (1–28) and FLAG-SIRT3 C2 (107–307) did not, suggesting that the 28–107 region is required for the interaction with NMNAT2. Among C-terminal cleavage fragments, SIRT3-C1 appeared to bear the highest affinity to Myc-NMNAT2, indicating that the region between residues 28–107 may be important for SIRT3-NMNAT2 interaction (Fig. 2B). We also tested the NMNAT2-SIRT3 interaction *in vitro* using purified SIRT3 proteins which were in agreement with our Co-IP results.

### SIRT3 deacetylates NMNAT2 under in vitro and in vivo assay conditions

To test whether SIRT3 deacelylated NMNAT2, in an acetylation buffer Flag-NMNAT2 was incubated with PCAF. Acetylation of the protein was determined by western blotting with antiacetyllysine antibody (Fig. 3A). Flag-NMNAT2 was acetylated *in vitro* with PACF and it was precipitated with Flag M2 beads. Acetylated Flag-NMNAT2 was then incubated with beads containing SIRT3 in a deacetylation buffer with or without NAD. SIRT3 was immunoprecipitated from stable A549 cells. This indicated that SIRT3 deacetylated of NMNAT2 *in vitro* is dependent on the NAD level (Fig. 3B and C). Stable cells expressing SIRT3 were induced to overexpress with Flag-NMNAT2 and treated with NAM (10 mM for 24 h) and/or TSA (5 *μ*M for 6 h) as indicated. Flag-NMNAT2 was immunoprecipitated and the level of acetylation was analyzed by probing with anti-acetyllysine antibody. It indicated that *in vivo* SIRT3 deacetylated NMNAT2 dependent on the TSA and NAM levels, especially related to TSA (Fig. 3D and E). Together, these data demonstrated that SIRT3 targets the enzyme NMNAT2, which catalyzes the formation of NAD (+) from nicotinamide mononucleotide (NMN) and ATP.

### Interaction of NMNAT2 with SIRT3 increases mitochondrial functions of A549 cells

To study the role interaction between SIRT3 and NMNAT2 on mitochondrial function, intact cellular basal oxygen consumption rates (OCR) of A549 cells were measured by Seahorse XF24 analyzer. The OCR of A549 cells transfected with NMNAT2 or NMNAT2+SIRT3 increased significantly compared to control (P<0.01), whereas, the OCR of A549 cells decreased significantly with SIRT3 interference (P<0.01) (Fig. 4A). Steady-state cellular ATP levels of A549 cells were also measured. The steady-state cellular ATP level of A549 cells transfected with NMNAT2 or NMNAT2+SIRT3 increased significantly compared to the A549 cells. The OCR of A549 cells decreased significantly (P<0.01) (Fig. 4B) with downregulation of SIRT3. There was significant expression of SIRT3 in NSCLC cell line A549. Adenovirus infection caused significant increase of SIRT3 in NSCLC cell lines. Transfection with SIRT1 siRNA caused reduction of protein after transfection (Fig. 4C). This suggested that SIRT1 siRNA selectively silences SIRT3 expression. NAD level of A549 cells transfected with NMNAT2 or NMNAT2+SIRT3 increased significantly compared to A549 cells. Downregulation of SIRT3, the OCR of A549 cells decreased significantly (P<0.01) (Fig. 5). The result showed that the interaction between NMNAT2 and SIRT3 promotes mitochondrial function levels of A549 cells.

### Interaction of NMNAT2 with SIRT3 promotes mitotic entry, cell growth and proliferation of A549 cells

To investigate the role of interaction between NMNAT2 and SIRT3 on mitotic entry, cell growth and proliferation, A549 cells were transfected with plasmids and synchronized at the G1/S transition as described in Materials and methods. Cells were pulse labeled with BrdU (50 *μ*M) for 30 min at indicated time-points after release from the second thymidine block. BrdU positive cells were detected by immunostaining and scored manually. More than 500 cells were counted in each of three independent experiments (Fig. 6A). Cell cycle progression of >1,000 cells was recorded by time-lapse videomicroscopy. The number of mitotic cells was scored by examination of individual cells (Fig. 6B). The results demonstrated that the interaction of NMNAT2 with SIRT3 promoted mitotic entry (Fig. 6). By XTT assays, we investigated the effect of the interaction between NMNAT2 and SIRT3 on cell growth and found that the growth of A549 cells transfected with NMNAT2 or NMNAT2+SIRT3 was more significant than in A549 cells (P<0.001). The growth of cells were significantly inhibited by interfering SIRT3 (P<0.001) (Fig. 7A). Cell viability was evaluated by CCK-8 assay. The result showed that the proliferation of A549 cells transfected with NMNAT2 or NMNAT2+SIRT3 was more significantly than in A549 cells (P<0.001). The growth of cells were significantly inhibited by interfering SIRT3 (P<0.001) (Fig. 7B). Our results indicated that the interaction of NMNAT2 with SIRT3 did not affect DNA synthesis, but low expression of SIRT3 significantly inhibited mitotic entry, growth and proliferation of A549 cells.

### Interaction of NMNAT2 with SIRT3 inhibits apoptosis of A549 cells

Our result showed that the apoptosis of A549 cells transfected with NMNAT2 or NMNAT2+SIRT3 was less than A549 cells (P>0.05). The apoptosis of cells were significantly promoted by interfering SIRT3 (P<0.001). This indicated that the interaction of NMNAT2 with SIRTs inhibited apoptosis of A549 cells (Fig. 8). Low expression of SIRT3 significantly promoted A549 cell apoptosis (the results from H1299 and PC-9 cells were similar to those from A549 cells).

## Discussion

NSCLC tumorigenesis follows a stepwise progression from hyperplasia to metaplasia, dysplasia, carcinoma *in situ* and, finally, to invasive tumors. To study the molecular pathogenesis of cancer during tumorigenesis, genes that inhibited lung carcinogenesis were identified. There are seven SIRT isoforms in mammals, with diverse biological functions including gene regulation, metabolism and apoptosis. SIRT3 is the primary mitochondrial deacetylase that modulates mitochondrial metabolic and oxidative stress regulatory pathways (10). However, its role in response to NSCLC remains unknown. In this study, we examined the role of SIRT3 in NSCLC.

At first, we investigated the novel SIRT3-interacting protein; we performed a yeast two-hybrid screening of a human lung cDNA library using full-length SIRT3 as a bait. Screening of transformants resulted in the isolation of several positive clones, which were identified encoding the full-length cDNA of NMNAT2 gene. We next examined the ability of SIRT3 protein to bind to NMNAT2 in yeast cells (Fig. 1A). These data demonstrated that SIRT3 interacts with NMNAT2 in yeast cells.

We examined the ability of SIRT3 protein to bind to NMNAT2 in mammalian cells. Our results showed a specific interaction between SIRT3 and NMNAT2 in NSCLC cells (Fig. 1B–D). To demonstrate the interaction of SIRT3 and NMNAT2 *in vitro*, GST pull-down assays were performed in which *in vitro* translated His-SIRT3 was incubated with full-length GST-NMNAT2 or Flag. As shown in Fig. 1E, SIRT3 interacted with GST-NMNAT2 but not with Flag alone (Fig. 1E). To test the colocalization, the cells were co-transfected with plasmids pEGFP-C1-SIRT3 and pDS-RED1-N1-NMNAT2. NMNAT2 (red, Fig. 1F) and SIRT3 (green, Fig. 1G) protein all localized to the cytoplasma. The overlaid images indicated that SIRT3 overlapped partly with NMNAT2 (Fig. 1I) in cytoplasma. These results indicate that SIRT3 interacted with NMNAT2 *in vivo* and *in vitro*. As shown in Fig. 2A, both full-length and the carboxy-terminal SIRT3 C1 fragments (residues 29–307) of SIRT3 protein interacted with Myc-NMNAT2. As shown in Fig. 2B, the results suggest that the 28–107 region is required for the interaction with NMNAT2. Among C-terminal cleavage fragments, SIRT3-C1 appeared to bear the highest affinity to Myc-NMNAT2, indicating that the region between residues 28–107 may be important for SIRT3-NMNAT2 interaction (Fig. 2B).

NMNAT2 belongs to the nicotinamide mononucleotide adenylyltransferase (NMNAT) enzyme family, members of which catalyze an essential step in the NAD (NADP) biosynthetic pathway. Unlike the other human family member, which is localized to the nucleus and is ubiquitously expressed; this enzyme is cytoplasmic and is predominantly expressed in the brain. Two transcript variants encoding different isoforms have been found for this gene (16). NMNAT2 is expressed predominantly in neurons (17–21). Its protein product has been shown to localize to the trans-Golgi complex (17,18), where it is packaged and transported down axons to the synapse (22). In addition to differences in tissue expression and intracellular localization, there is an isofrom specific domain on each of the NMNAT genes (23). In NMNAT2 this region is palmitoylated at two cysteine residues and, when cleaved, the NAD^+^ synthesis activity of the enzyme increases significantly (18,24). This provides a mechanism to increase the cytosolic pool of NAD^+^ quickly in response to a stimulus such as cell stress. We tested our hypothesis that SIRT3 deacetylated NMNAT2. Our study showed an association of NMNAT2 with SIRT3 suggesting that NMNAT2 is the deacetylation target of SIRT3, which had the ability to deacetylate NMNAT2 in an NAD-dependent manner (Fig. 3). NMNAT2 was highly acetylated in cells treated with the HDAC inhibitors TSA and NAM compared to non-treated controls. When NMNAT2 was analyzed from SIRT3-expressing cells, we found that it was substantially deacetylated in these cells but not in cells expressing SIRT3. These data thus indicated that SIRT3 is one of the major regulators of NMNAT2 acetylation *in vivo*.

SIRT3 was the only sirtuin implicated in extension of life span in human (25) and recent evidence has shown its involvement in mitochondrial energy metabolism and biogenesis (26) and preservation of ATP biosynthetic capacity in the heart (26). SIRT3 was shown to regulate the activity of acetyl-CoA synthetase 2 (AceCS2), an important mitochondrial enzyme involved in generating acetyl-CoA for the tricarboxylic acid (TCA) cycle. In these studies, SIRT3 knockout resulted in a marked decrease of basal ATP level *in vivo* (27). Recent studies in cardiomyocytes demonstrated the protective role of SIRT3 from oxidative stress and hypertrophy (28,29). Accordingly, the evidence suggests that SIRT3 could also have a pivotal role in protecting neurons from injury due to conditions that promote bioenergetic failure, such as excitotoxicity. Mitochondrial localization of SIRT3 plays a role in various mitochondrial functions, such as maintaining basal ATP level and regulating apoptosis. SIRT3 has been shown to regulate energy homeostasis (26). As a critical factor in energy metabolism for cell survival, nicotinamide adenine dinucleotide (NAD) has drawn considerable interest. NAD is an essential molecule playing a pivotal role in energy metabolism, cellular redox reaction and mitochondrial function. Recent studies have revealed that maintaining intracellular NAD is important in promoting cell survival in various types of diseases, including axonal degeneration, multiple sclerosis (MS), cerebral ischemia and cardiac hypertrophy (28,30–39). Loss of NAD decreases the ability of NAD-dependent cell survival factors to carry out energy-dependent processes, leading to cell death.

In this study, we identified NMNAT2 as a new target of SIRT3 deacetylase. NMNAT2 is found in mitochondria and identified to target SIRT3. The function of the interaction between SIRT3 and NMNAT2 have been identified. The results showed that the interaction of NMNAT2 with SIRT3 increases mitochondrial functions of A549 cells (Figs. 4 and 5). the roles of SIRT3 and NMNAT2 on NSCLC cell lines related to energy metabolism were associated with the interaction between SIRT3 and NMNAT2. Moreover, the interaction of NMNAT2 with SIRT3 promoted mitotic entry, cell growth and proliferation of A549 cells and inhibited apoptosis of A549 cells (Figs. 6–8).

Lung cancer is the leading cause of cancer-related mortality in the worldwide, which is the third most common malignant disease and ∼75% of all diagnosed lung cancers are non-small cell lung carcinoma (NSCLC) and is associated with dismal prognoses. Chemotherapy in addition to surgical resection and radiotherapy remains a basic strategy for treatment of malignant tumors. Unfortunately, it has been shown that NSCLC only has a limited sensitivity to chemotherapeutic drugs. A major obstacle in the treatment of patients is the inherent resistance to chemotherapeutic agents. Inhibition of cell apoptosis pathway was reported as one important cellular mechanism responsible for the resistance of NSCLC cells to treatment.

Thus, our results strongly suggest that the binding of SIRT3 with NMNAT2 is a novel regulator of cell proliferation and apoptosis in NSCLC cell lines implicating the interaction between SIRT3 and NMNAT2 and energy metabolism associated with it. This study demonstrates that the interaction between SIRT3 and NMNAT2 may be a novel opportunity for future research for treatment of NSCLC.

## Figures and Tables

**Figure 1.** NMNAT2 interacts with SIRT3 in yeast, in mammalian cells and *in vitro*. (A) Identification of NMNAT2 as a SIRT3-interacting protein by the yeast two-hybrid assay. Yeast AH109 cells were transformed with different plasmids and grown on SD/-Trp-Leu-His-Ade. +, grown within 96 h; −, no growth within 96 h. Positive colonies were tested for β-galactosidase activity. +, turned blue within 2 h; −, did not turn blue within 2 h. (B) Interaction of NMNAT2 with SIRT3 in mammalian cells. A549 cells, cultured in regular medium, were transfected with expression plasmids as indicated. Immunoprecipitation (IP) and immunoblotting (IB) were performed using anti-FLAG or anti-Myc monoclonal antibody respectively. (C) To test NMNAT2 interacting with SIRT3 *in vivo* by Mammalian Two-Hybrid system. A549 cells were transfected with expression plasmids as indicated and cultured in regular medium. At 48 h after transfection, cells were evaluated by firely luciferase assays. Significance was determined on the mean of three different experiments. The luciferase levels of pACT-NMNAT2 and pBIND-SIRT3 were ≥2.64 times higher than negative control (P<0.05). These results indicate that NMNAT2 interacted with SIRT3 *in vivo* and *in vitro*. Values are means of three experiments. All data are presented as the mean ± SEM. (D) The expressing of NMNAT2 and SIRT3 in lysate of the cells. The lysates of A549 cells transfected with those plasmids were detected by IB with anti-NMNAT2 and anti-SIRT3 monoclonal antibody. (E) Interaction of SIRT3 with NMNAT2 *in vitro*. Glutathione-Sepharose beads bound with FLAG-SIRT3 or with FLAG were incubated with His-NMNAT2. After washing the beads, the bound proteins were eluted and subjected to SDS-PAGE and autoradiography. To demonstrate the colocalization of NMNAT2 and SIRT3 in A549 cells, they were cultured, then co-transfected with plasmids. After 48 h, cells were stained with PFA and DAPI; confocal images were acquired using Zeiss 510 META confocal microscope. NMNAT2 protein (red) localized to the cytoplasma (F). SIRT3 (green) localized in the cytoplasma (G). The nuclear of cells (blue) were stained by DAPI (H). The overlaid images indicated that NMNAT2 overlapped partly with SIRT3 in the cytoplasma (I).

**Figure 2.** Map of the NMNAT2 and SIRT3 interaction regions. (A) Mapping of SIRT3 interaction region in NMNAT2. (B) Co-immunoprecipitation of NMNAT2 and SIRT3. Map of the NMNAT2 SIRT3-interacting domains. Myc-SIRT3 and NMNAT2-Flag and its derivatives were overexpressed in A549 cells. NMNAT2-Flag protein was pulled down by Protein G Plus/Protein A Agarose Suspension beads. The presence of SIRT3 was detected by Myc immunoblotting.

**Figure 3.** SIRT3 deacetylates NMNAT2 under *in vitro* and *in vivo* assay conditions. (A) In an acetylation buffer Flag-NMNAT2 was incubated with PCAF and acetylation of protein was determined by western blotting with antiacetyllysine antibody. (B) Deacetylation of NMNAT2 by SIRT3 *in vitro*. Flag-NMNAT2 was acetylated *in vitro* with PACF and it was precipitated with Flag M2 beads. Acetylated Flag-NMNAT2 was then incubated with beads containing SIRT3 in a deacetylation buffer with or without NAD. SIRT3 was immunoprecipitated from stable A549 cells. (C) Quantification of NMNAT2 deacetylation by SIRT3. (D) *In vivo* deacetylation of NMNAT2 by SIRT3. Stable cells expressing SIRT3 were induced to overexpress with Flag-NMNAT2 and treated with NAM (10 mM for 24 h) and/or TSA (5 *μ*M for 6 h) as indicated. Flag-NMNAT2 was immunoprecipitated and the level of acetylation was analyzed by immunoblotting with antiacetyllysine antibody. (E) Quantification of NMNAT2 deacetylation by SIRT3 *in vivo*. Values are means of three experiments. All data are presented as the mean ± SEM.

**Figure 4.** Interaction of NMNAT2 with SIRT3 boosted strongly mitochondrial functions of A549. Intact cellular basal oxygen consumption rates (OCR) of A549 cells were measured by Seahorse XF24 analyzer. The OCR of A549 cells transfected with NMNAT2 or NMNAT2+SIRT3 increased significantly compare to A549 cells (P<0.01). SIRT3 interference decreased significantly the OCR of A549 cells (A) (P<0.01). The steady-state cellular ATP level of A549 cells transfected with NMNAT2 or NMNAT2+SIRT3 increased significantly compared to A549 cells, whereas, downregulation of SIRT3, decreased the OCR significantly in A549 cells (B) (P<0.01). Adenovirus infection caused significant increase of SIRT3 in NSCLC cell lines. Transfection with SIRT3 siRNA caused reduction of proteins after 48 h (C). Values are the means of three experiments. All data are presented as the mean ± SEM.

**Figure 5.** Interaction of NMNAT2 with SIRT3 increases NAD levels of A549. NAD level of A549 cells transfected with NMNAT2 or NMNAT2+SIRT3 was more significant than in the A549 cells alone. Downregulation of SIRT3, decreased significantly (P<0.01) the OCR of A549 cells. Values are the means of three experiments. All data are presented as the mean ± SEM.

**Figure 6.** Interaction of NMNAT2 with SIRT3 promotes mitotic entry of A549. (A) Interaction of NMNAT2 with SIRT3 did not affect DNA synthesis. A549 cells were transfected with plasmids and synchronized at the G1/S transition as described in Materials and methods. Cells were pulse-labeled with BrdU (50 *μ*M) for 30 min at indicated time-points after release from the second thymidine block. BrdU positive cells were detected by immunostaining and scored manually. More than 500 cells were counted in each of the three experiments. (B) Interaction of NMNAT2 with SIRT3 promoted mitotic entry. Cell cycle progression of >1,000 cells was recorded by time-lapse videomicroscopy. The number of mitotic cells was scored by examination of individual cells. Values are means of three experiments. All data are presented as the mean ± SEM.

**Figure 7.** Interaction of NMNAT2 with SIRT3 promoted mitotic growth and proliferation of A549 cells. (A) By XTT assays, we investigated the effect of the interaction between NMNAT2 and SIRT3 on cell growth and found that the growth of A549 cells transfected with NMNAT2 or NMNAT2+SIRT3 was more significant than in A549 cells (P<0.001). The growth of cells were significantly inhibited by interfering SIRT3 (P<0.001). (B) Cell viability was evaluated by CCK-8 assay. The result showed that the proliferation of A549 cells transfected with NMNAT2 or NMNAT2+SIRT3 was more significant than in A549 cells (P<0.001). The growth of cells were significantly inhibited by interfering SIRT3 (P<0.001). Values are means of three experiments. All data are presented as the mean ± SEM.

**Figure 8.** Interaction of NMNAT2 with SIRT3 inhibited apoptosis of A549 cells. The result showed that the apoptosis of A549 cells transfected with NMNAT2 or NMNAT2+SIRT3 was less than in A549 cells (P>0.05). The apoptosis of cells were significantly promoted by interfering SIRT3 (P<0.001). Values are means of three experiments. All data are presented as the mean ± SEM.
